This article has been retracted.

# Mortality Risk Factors for Patients With Sepsis-Induced Blood Pressure Drop: A Single-Center Retrospective Study

**DOI:** 10.7759/cureus.22114

**Published:** 2022-02-11

**Authors:** Vicky Kumar, Sabeen Sharif Khan, Yousef Awad, Zahoor Ur Reham, Fares Mohammed Saeed Muthanna, Ellen Huang, Marina Basta, Hajra Khwaja, Rahil Barkat

**Affiliations:** 1 Internal Medicine, South City Hospital, Irbid, JOR; 2 Medicine, Aga Khan University Hospital, Karachi, PAK; 3 Clinical Research, The Oncology Institute of Hope and Innovation, Cerritos, USA; 4 Internal Medicine, Al Rahba Hospital, Abu Dhabi, ARE; 5 Pharmaceutical Care, Walailak University, Nakhon Si Thammarat, THA; 6 Internal Medicine, Oceania University of Medicine, Apia, WSM; 7 School of Medicine, St. George's University, True Blue, GRD; 8 Research Department, Aga Khan University Hospital, Karachi, PAK; 9 Indus Hospital Research Center, The Indus Hospital, Karachi, PAK

**Keywords:** induced, frequency, risk factors, blood pressure, sepsis

## Abstract

Introduction: Sepsis is a life-threatening illness caused by the body's response to uncontrolled infection. Different studies have been conducted to identify risk factors associated with the diagnosis of sepsis and mortality, but there has been considerably less focus on mortality due to sepsis-induced blood pressure. The current study was conducted to determine the incidence of mortality within 30 days among patients with sepsis-induced blood pressure drop and its risk factors.

Methodology: It was a retrospective study conducted at the Pakistan Navy Station (PNS) Shifa Hospital, Karachi, Pakistan. Data of all patients aged 18 years or more who visited PNS Shifa Hospital and were diagnosed with sepsis and blood pressure reduction from November 2019 to October 2021 were extracted from Hospital Management Information System (HMIS) and retrospectively analyzed

Results: All variables significantly associated with 30-days mortality in multivariable logistic regression analysis, including disturbance of consciousness, cardiac insufficiency, respiratory failure, diabetes mellitus, creatinine level, and aspartate aminotransferase (AST) level, were risk factors for mortality in patients with the sepsis-induced drop in blood pressure (p-value<0.05).

Conclusion: Identifying these risk factors is important as it will help clinicians identify patients who are at high risk of mortality at an early stage. Through early identification, interventions can be done to reduce the incidence of in-hospital mortality among sepsis patients.

## Introduction

Sepsis is a life-threatening illness caused by the body's response to uncontrolled infection. It affects millions of individuals each year across the world [1]. In the United States, septicemia is the eleventh leading cause of death [2]. A study conducted on hospitalized patients in the United States showed that sepsis increases by almost 8% every year [3]. Besides this, more than half of all hospital deaths are caused by sepsis, signifying the burden of sepsis on human health and the healthcare system [4].

Different studies have been conducted to identify risk factors associated with a diagnosis of sepsis and mortality, but there has been considerably less focus on mortality due to sepsis-induced blood pressure drop. Few studies have addressed how these patients need to be treated and the risk factors associated with it for the development of predictive tools [5,6]. Sepsis, which is caused by infection, frequently causes immune system problems as well as clinical signs such as heart, kidney, and coagulation failure, raising the risk of death [7]. Furthermore, patients with sepsis-induced blood pressure drop have hypoperfusion symptoms. Blood pressure reduction owing to sepsis is linked to poor clinical outcomes, according to actual experience in clinical practice [8]. Because this pathology is more life-threatening than sepsis alone, a study of this cohort would be extremely valuable.

Currently, similar scoring techniques such as the Acute Physiology and Chronic Health Evaluation II (APACHE-II) or the Sequential Organ Failure Assessment score (SOFA score) are used in the clinical evaluation of the severity and mortality estimation in patients with sepsis-induced blood pressure drop [9]. These scores have certain limitations in the assessment of patients with sepsis-induced blood pressure drop. For instance, APACHE II can only be used in critically ill patients. In addition, SOFA can be used for the prediction of multiple organ dysfunction syndrome [8]. The current study can help to identify risk factors associated with mortality in the short term of patients with sepsis-induced blood pressure drop.

It is important to identify patients at high risk of mortality due to sepsis-induced blood pressure drop to intervene early and reduce the incidence of mortality among sepsis patients in hospital settings. No previous studies have been conducted in Pakistan regarding the identification of risk factors of mortality due to sepsis-induced blood pressure drop. Therefore, the current research has been conducted to determine the incidence of mortality within 30 days among patients with sepsis-induced blood pressure drop and risk factors associated with it.

## Materials and methods

Methodology

It was a retrospective study conducted at the Pakistan Navy Station (PNS) Shifa Hospital, Karachi, Pakistan. Data of all patients aged 18 years or older, who visited PNS Shifa Hospital and were diagnosed with sepsis and blood pressure reduction from November 2019 to October 2021 were extracted from the Hospital Management Information System (HMIS) and retrospectively analyzed.

Patients with human immunodeficiency autoimmune diseases, aplastic anaemia, liver cirrhosis, and leukaemia were excluded from the study. Moreover, patients with pancreatitis, primary peritonitis, and other shocks, including hypotension due to analgesic drugs, allergic reaction to medication usage in an emergency room, or with other diseases at the time of admission, were also excluded from the study. Data of patients who left the hospital without improvement in clinical conditions within 30 days were not included in the final analysis, along with patients who left without medical advice and shifted to another hospital. Lastly, patients with missing data (outcome data is missing) were not included in the final analysis.

Outcome variable

Whether the outcome was "death" or "survivor" was determined from the HMIS as recorded when patients were discharged from the hospital. If a patient died in the hospital, the outcome was categorized as death. On the other hand, if a patient left the hospital with improvement in clinical conditions, the outcome will be categorized as a survivor.

For the purpose of this study, sepsis was defined as organ dysfunction activated by an infection that puts the patient’s life in danger. A rapid increase in the SOFA score with a total of 2 pointsis an indicator of organ failure [8]. A systolic blood pressure drop of 40 mm Hg from the original basal blood pressure or from normal blood pressure, or a systolic blood pressure of less than 90 mm Hg at the time of admission to the wards, were used to evaluate blood pressure reduction [8].

Independent variables

Following variables were collected: age, sex, BMI, comorbidities, and laboratory values at the time of admission, including the number of WBCs (10*9/L), number of platelets (10*9/L), haemoglobin level (g/dl), creatinine level (mmol/L), C-reactive protein (mg/L), total bilirubin (umol/L), albumin level (g/L), sodium concentration (mmol/L), potassium concentration (mmol/L), alanine transaminase (IU/L) and aspartate transaminase (IU/L). Other variables included consciousness disturbance (defined as whether a patient was in coma, lethargic, or drowsy), heart function (considering the classification of New York Heart Association, that is cardiac function class III or above) [10] and respiratory failure (concentration of oxygen <=300 mm Hg) at the time of admission.

Statistical analysis

All the analysis was done on Stata Statistical Software: Release 16 (2019; StataCorp. LLC, College Station, Texas). Descriptive statistics were presented as mean and standard deviation for continuous variables, including age, frequency, and percentages, were calculated for categorical variables. Laboratory values were presented as a median and interquartile range, and a comparison of laboratory values between survivors and dead patients was done using the Mann-Whitney U test. The chi-square test was used to assess categorical variables between two groups. Potential risk factors for mortality were evaluated by univariate analysis, and factors with p-values <0.05 were included in a multivariable model. Multivariable logistic regression was used to control the confounding factors, and P <0.05 was considered to indicate statistical significance.

## Results

From November 2019 to October 2021, a total of 892 patients with sepsis and blood pressure reduction visited the hospital. Out of these, 292 patients did not fulfill the eligibility criteria and the data of another 67 patients were missing. Hence, a total of 533 patients were included in the study. The demographic characteristics of the patients are shown in Table 1. The mean age of the participants was 67.83 +/- 16.49 years. The majority of participants were males (58.16%) and had normal BMI (52.16%). Mortality within 28 days was reported in 19.89% of patients.

**Table 1:** Demographic characteristics of patients * Mean (SD) BMI: body mass index

Variable	Categories	n (%)
Age*		67.83 +/- 16.49
Sex	Male	310 (58.16)
	Female	223 (41.84)
Mortality	No	427 (80.11)
	Yes	106 (19.89)
BMI	Underweight	53 (9.94)
	Normal	278 (52.16)
	Overweight	112 (21.01)
	Obese	90 (16.88)

Table 2 shows the comparison of demographic and clinical characteristics of the patients who died and those who survived. Age was significantly higher among the patients who died (72.95 +/- 1.25) as compared to the survivors (66.55 +/- 17.07) (p-value=0.003). The proportion of disturbance of consciousness was significantly lower in the survivor group as compared to patients who died (p-value=0.001). Additionally, respiratory failure and cardiac insufficiency were also lower in the survivor group than patients who died (p-value<0.05). In relation to comorbidity, only diabetes was significantly different in the two groups; diabetes was present in more patients who died (47.17%) than in the survivors (40.28%) (p-value=0.001).

**Table 2:** Comparison of characteristics between groups ^ Mean (Standard deviation); * Significant at p-value<0.05 BMI: body mass index; CHD: coronary heart disease

Variables	Categories	Mortality		p-value
		No n (%)	Yes n (%)	
Age^		66.55 +/- 17.07	72.95 +/- 1.25	0.003*
Sex	Male	243 (56.91)	67 (63.21)	0.239
	Female	184 (43.09)	39 (36.79)	
BMI	Underweight	45 (10.54)	8 (7.55)	0.255
	Normal	220 (51.52)	58 (54.72)	
	Overweight	93 (21.77)	19 (17.92)	
	Obese	69 (16.16)	21 (19.81)	
Disturbance of consciousness	No	346 (81.03)	57 (53.77)	0.001*
	Yes	81 (18.97)	49 (46.23)	
Cardiac Insufficiency	No	368 (86.18)	63 (59.43)	0.001*
	Yes	59 (13.82)	43 (40.57)	
Respiratory failure	No	355 (83.14)	52 (49.06)	0.001*
	Yes	72 (16.86)	54 (50.94)	
Comorbidities				
Hypertension		235 (55.04)	73 (68.87)	0.011*
Diabetes mellitus		172 (40.28)	50 (47.17)	0.198
CHD		95 (22.25)	21 (19.81)	0.586
Other		129 (30.21)	35 (33.02)	0.575

Table 3 shows the laboratory values in two groups. Laboratory values were significantly different in two groups including platelets (p-value=0.001), creatinine (p-value=0.001), C-reactive protein (p-value=0.022), albumin (p-value=0.001), potassium (p-value=0.002), alanine transaminase (ALT) (p-value=0.001), and aspartate aminotransferase (AST) (p-value=0.001).

**Table 3:** Comparison of laboratory values between groups * Significant at p-value<0.05; Presented as Median (interquartile range) WBC: white blood cells; CRP: C-reactive protein; ALT: alanine transaminase; AST: aspartate transaminase

Variables	Mortality		p-value
	No	Yes	
WBC (10*9/L)	10.4 (6.3-16)	12.15 (6.5-17.9)	0.166
Platelets (10*9/L)	136 (87-199)	96.5 (59-177)	0.001*
Hemoglobin (g/dl)	11.5 (10.9-12.1)	11.8 (11.0-12.6)	0.544
Creatinine (mmol/L)	80 (61-134)	124 (71-212)	0.001*
CRP (mg/L)	102.10 (57.33-169.90)	125.65 (61.99-200)	0.022*
Total bilirubin (umol/L)	10.7 (7.3-16.7)	12.2 (7.4-26.3)	0.076
Albumin (g/L)	29.6 (26.3-32.5)	26.6 (23.9-30.6)	0.001*
Sodium (mmol/L)	136 (133-139)	135 (133-137)	0.181
Potassium (mmol/L)	4.2 (3.9-4.5)	4.5 (4.0-4.9)	0.002*
ALT (IU/L)	32 (23-41)	44.5 (15-55)	0.001*
AST (IU/L)	31 (24-45)	55 (37-63)	0.001*

All variables that were significantly associated with 30-days mortality at univariate analysis were tested at multivariable logistic regression analysis. Variables significantly associated with the outcome are shown in Table 4. Disturbance of consciousness, cardiac insufficiency, respiratory failure, diabetes mellitus, creatinine level, and AST level were found to be risk factors for mortality in patients with the sepsis-induced drop in blood pressure (p-value<0.05).

**Table 4:** Variables that were found to be significantly associated with mortality (multivariable logistic regression) AOR (Adjusted odds ratio); AST: aspartate aminotransferase

Variable	Categories	AOR (95% CI)	p-value
Disturbance of consciousness	No		
	Yes	3.76 (1.90-7.44)	0.001
Cardiac insufficiency	No		
	Yes	2.26 (1.13-4.52)	0.002
Respiratory failure	No		
	Yes	6.70 (3.42-13.11)	0.001
Diabetes mellitus	No		
	Yes	2.60 (1.37-4.92)	0.003
Creatinine level		1.01 (1.00-1.02)	0.005
AST		1.02 (1.01-1.03)	0.001

## Discussion

The current study was conducted to determine the incidence and risk factors associated with 30-days mortality due to sepsis-induced blood pressure drop. The current study showed that mortality within 30 days due to sepsis-induced blood pressure drop was reported in 19.89% of patients. As per the study conducted by Wang and Chen, the death rate within 30 days due to sepsis-induced blood pressure drop was found to be 20.7% of patients [5]. Our study has found that risk factors associated with 30-days mortality included disturbance of consciousness, cardiac insufficiency, respiratory failure, estimated glomerular filtration rate (eGFR), diabetes mellitus, creatinine level, and AST level.

Our results showed that cardiac insufficiency is a death-related risk factor as found in a previous study [11]. In patients with sepsis-induced blood pressure drop, the treatment needs fluid resuscitation. On the other hand, for patients with cardiac insufficiency and heart dysfunction, improper fluid resuscitation and increased fluid sensitivity can increase the risk of death [12]. 

It is believed that patients with respiratory failure will suffer from hypoxia, and it will increase the risk of death. Sepsis involves a multifaceted interaction between the inflammatory and coagulation systems at the microvascular and endothelial level, leading to tissue hypoperfusion and, therefore, inducing hypoxia [13]. Even if patients are treated with a ventilator, complications in the treatment can also lead to increased mortality [14]. Our study has shown that patients with respiratory failure are at a higher risk of death. Therefore, it should be considered as an important risk factor while treating patients with sepsis-induced blood pressure drops in order to decrease the chance of mortality.

Another factor highlighted in the current study is a disturbance of consciousness. Patients with disturbance of consciousness are at higher risk of mortality. Consciousness disturbance means the decrease of self-protection function that can cause certain complications, including asphyxia, and also results in mortality [5]. This study's findings are supported by the study conducted by Wang and Chen [5]. Creatinine level is the most commonly used index to assess renal function and patients with poor renal function are at higher risk of mortality [15]. The current study has found that increased creatinine level is one of the important risk factors of mortality due to sepsis-induced blood pressure drop.

In our study, diabetes was also one of the significant factors associated with in-hospital mortality. The study conducted by Drumheller et al., in their retrospective, single-centre observational cohort study of severe sepsis and septic shock patients in an emergency department, found that diabetes mellitus is independently associated with in-hospital mortality among septic patients [16].

The current study has certain limitations. Firstly, it is a retrospective study; therefore, we were unable to assess different risk factors, including smoking status, lactate levels, and procalcitonin, which are important indicators of mortality but were not recorded in medical records of patients. Secondly, it was a single-centred study, therefore, lacking verification of data with several other tertiary care hospitals. In the future, further prospective studies need to be conducted considering all clinical and non-clinical indicators to identify risk factors associated with mortality among patients with sepsis-induced blood pressure drop. Identification of these risk factors is important to identify patients who are at increased risk of mortality in order to provide them with early interventions.

## Conclusions

The study determined the incidence of mortality within 30 days among patients with sepsis-induced blood pressure drop and risk factors associated with it. The study found that disturbance of consciousness, cardiac insufficiency, respiratory failure, eGFR, diabetes mellitus, creatinine level, and AST level is associated with 30-days mortality in patients with sepsis-associated blood pressure drop. Identifying these risk factors is important as it will help clinicians in identifying patients at an early stage who are at high risk of mortality, thus reducing the incidence of in-hospital mortality among sepsis patients.

## References

[1] Degoricija V, Sharma M, Legac A, Gradišer M, Šefer S, Vučičević Ž (2006). Survival analysis of 314 episodes of sepsis in medical intensive care unit in university hospital: impact of intensive care unit performance and antimicrobial therapy. Croat Med J.

[2] Kochanek KD, Xu J, Murphy SL, Miniño AM, Kung HC (2011). Deaths: preliminary data for 2009. Natl Vital Stat Rep.

[3] Fleischmann C, Scherag A, Adhikari NK (2016). Assessment of global incidence and mortality of hospital-treated sepsis. Current estimates and limitations. Am J Respir Crit Care Med.

[4] Zhou J, Qian C, Zhao M (2014). Epidemiology and outcome of severe sepsis and septic shock in intensive care units in mainland China. PLoS One.

[5] Wang B, Chen J (2021). Establishment and validation of a predictive model for mortality within 30 days in patients with sepsis-induced blood pressure drop: A retrospective analysis. PLoS One.

[6] Bijker JB, van Klei WA, Kappen TH, van Wolfswinkel L, Moons KG, Kalkman CJ (2007). Incidence of intraoperative hypotension as a function of the chosen definition: literature definitions applied to a retrospective cohort using automated data collection. Anesthesiology.

[7] Lambden S, Creagh-Brown BC, Hunt J, Summers C, Forni LG (2018). Definitions and pathophysiology of vasoplegic shock. Crit Care.

[8] Vincent JL, Moreno R, Takala J (1996). The SOFA (Sepsis-related Organ Failure Assessment) score to describe organ dysfunction/failure. On behalf of the Working Group on Sepsis-Related Problems of the European Society of Intensive Care Medicine. Intensive Care Med.

[9] Baykara N, Akalın H, Arslantaş MK (2018). Epidemiology of sepsis in intensive care units in Turkey: a multicenter, point-prevalence study. Crit Care.

[10] Fisher JD (1972). New York Heart Association classification. Arch Intern Med.

[11] Ng PY, Sin WC, Ng AK, Chan WM (2016). Speckle tracking echocardiography in patients with septic shock: a case control study (SPECKSS). Crit Care.

[12] HE L (2018). Application value of PICCO and CVP monitoring in treatment of patients with septic shock complicated with cardiac insufficiency. J Jilin Univ Med Ed.

[13] van der Poll T, de Boer JD, Levi M (2011). The effect of inflammation on coagulation and vice versa. Curr Opin Infect Dis.

[14] Song JE, Kim MH, Jeong WY (2016). Mortality risk factors for patients with septic shock after implementation of the surviving sepsis campaign bundles. Infect Chemother.

[15] Perrone RD, Madias NE, Levey AS (1992). Serum creatinine as an index of renal function: new insights into old concepts. Clinical chemistry.

[16] Drumheller BC, Agarwal A, Mikkelsen ME, Sante SC, Weber AL, Goyal M, Gaieski DF (2016). Risk factors for mortality despite early protocolized resuscitation for severe sepsis and septic shock in the emergency department. J Crit Care.

